# Study on the Effect of Driving Time on Fatigue of Grassland Road Based on EEG

**DOI:** 10.1155/2021/9957828

**Published:** 2021-07-08

**Authors:** Yule Zhang, Shoulin Zhu

**Affiliations:** College of Energy and Transportation Engineering, Inner Mongolia Agricultural University, Hohhot 010000, China

## Abstract

In order to study the change law of the fatigue degree of grassland expressway drivers over time, this paper takes the semidesert grassland landscape of Xilinhot city as the experimental environment and takes the provincial highway S101 (K278–K424) as an example to design an actual driving test. Taking Urumqi, Inner Mongolia Autonomous Region, as the experimental section, combined with the Biopac MP150 multichannel physiological instrument and its auxiliary knowledge software and mathematical statistics methods, the relationship between EEG and time was studied. The test results show that the primary fatigue factor *F*_1_ and the secondary fatigue factor *F*_2_ can summarize the fatigue law characterized by 96.42% of EEG information. During 130 minutes of driving on the prairie highway, the periods of high fatigue were 105 minutes and 125 minutes, respectively. Driving fatigue can be divided into three stages over time: 5–65 min fatigue-free stage, 70–85 min fatigue transition stage, and 90–130 min fatigue stage. Fatigue changes over time. The law follows the Gaussian function and the sine function.

## 1. Introduction

Drivers need to keep their concentration in the road environment to ensure the safety of driving tasks [1]. Studies have shown that low load conditions such as monotony can lead to fatigue symptoms and impaired driving performance, although drivers are neither tired nor lack sleep before driving tasks [2, 3]. This kind of fatigue is caused by driving itself, which is called passive fatigue. Passive fatigue is caused by nerve habituation, such as driving on similar and repeated routes [4], which is different from the driver's active fatigue caused by physiological rhythm and lack of sleep [5]. Fell and Black conducted a driver fatigue accident survey in Sydney, which covered all accidents caused by fatigue. It was found that 45% of crash drivers were not tired at all before the accident, and the road geometry was very monotonous [6]. It can be seen that the accidents caused by driving fatigue in the monotonous environment are potential. The research on this kind of fatigue can effectively reduce the accident rate. Relevant research shows that the most reliable way to quantify driver mental fatigue in the monotonous environment is to use electroencephalogram (EEG), which is a very promising indicator [7].

The influencing factors of driving fatigue include not only the monotonous degree of the road environment, the physiological rhythm of drivers, and the time of driving but also the duration of work. Driving for a long time will increase the fatigue degree. Research shows that 30 minutes of monotonous driving can cause alertness disorder [8], 11% of accidents are related to fatigue, and 62% of accidents occur in driving less than 100 miles, that is, 87.6 minutes [4]. Larue et al. proposed that the effect of quantitative time on fatigue needs to be set beyond 40 minutes [9]. Therefore, in the monotone road environment, the time task test of more than one hour is the basis of quantifying the effect of time on fatigue.

The mileage of roads in the Inner Mongolia Autonomous Region is increasing constantly. By the end of 2018, the total mileage of class roads was 192,200 kilometers, of which grassland roads accounted for 73.3%. Grassland road has the characteristics of monotonous roadside landscape and road alignment. When driving on prairie roads, drivers will encounter the problem of insufficient stimulus information, which will easily lead to the decrease of driver's attention and alertness, premature driving fatigue, and traffic accidents [10].

The innovative content of this paper is as follows:

1. Combining the Biopac MP150 multichannel physiological instrument and its auxiliary knowledge software and mathematical statistics methods, the relationship between EEG and time has been studied
2. The EEG model is used to analyze and research related fatigue data
3. The EEG model and EEG are used to study the relationship between driving fatigue and fatigue data

## 2. Materials and Methods

### 2.1. Test Personnel

In the experimental study, the number and representativeness of the subjects will directly affect the reliability of the experimental results. In formula (1), *n* is the required sample size [11], *Z* is the statistics with a certain confidence level, and *s* is the standard deviation of each test index of driving characteristics [12]. Based on the research results at home and abroad, *s* = 0.094 and *d* = 0.04; in this paper, *z* = 1.96 at 95% confidence level is taken; the minimum number of subjects in this experimental study is 22. Taking into account the characteristics of significant individual differences in EEG signals and susceptibility to environmental factors, the number of subjects was determined as 30 in this experiment.

(1) $$\begin{array}{c} n\geq \frac{z^{2}\times s^{2}}{d^{2}}. \end{array}$$

According to the statistics that the proportion of male and female drivers with legal driving license is 7/3 and the analysis of driving age and age of drivers in traffic accidents [13], the test subjects are determined, as shown in Table 1.

In order to ensure the effectiveness of data collection, the requirements for the test driver are as follows: good health, sufficient sleep before the test, no activities that stimulate the heart within 24 hours, no smoking, and vigorous exercise 1 hour before the test.

### 2.2. Road Sections and Test Vehicles

The test section is S101 provincial road in Xilinhot city, Inner Mongolia. The relevant parameters of the section are shown in Table 2: 84.9% of the road lines are long straight lines, with large curve radius and 61% of large radius curves. The longitudinal slope is gentle, and the undulation is not obvious. In addition, the vegetation coverage is low, and the desertification is serious. The test section has the characteristics of monotonous landscape and line type.

By the end of 2017, China's car ownership was 209.0667 million, including 180.3869 million small passenger vehicles, accounting for 86.28% (China National Bureau of statistics, http://data.stats.gov.cn/index.htm). The research group investigated the traffic flow of the grassland road, and the proportion of small vehicles was 91.5%. Therefore, the Honda Civic car (automatic transmission) is used as the test vehicle. According to the time task test, the time of the vehicle to be tested must be more than 40 min. The test road section is selected to be 150 km long in one way, 300 km back and forth, and 150 min under the speed limit of 80 km/h.

### 2.3. Test Process

The choice of test time and the control of the environment will seriously affect the test results. In order to reduce the influence of factors other than time on the results, sunny days with similar illuminance and postlunch dip were selected for testing [14], which was the peak period of daytime fatigue accidents. The subjects arrived at the test site at 12:30. Familiar with the test equipment, understand the test requirements, complete the wiring work; 12:50, drive for 5 minutes, familiar with the environment and equipment; 13:00, officially start the test.

### 2.4. Test Instruments and Requirements

The MP150 multichannel physiological recorder (maximum sampling rate: 400 kHz, including the EEG amplifier) and AcqKnowledge 4.1 data analysis software are used to obtain the EEG data. The research related to the fatigue of monotonous road drivers is to characterize the driver's mental fatigue by the average power of three waveforms of *α* (8–13 Hz), *β* (14–30 Hz), and *θ* (4–7 Hz). The sampling frequency is adjusted to 250 Hz based on kurtosis and probability criteria, and the band-pass filter frequency is set to 1 Hz (high-pass filter) to 30 Hz (low-pass filter) [15]. Two lead 110 shield wires are, respectively, connected to the disposable electrode piece on the driver's left forehead and right mastoid, and the other end is connected to the EEG100C EEG amplifier (the amplifier gain is set at 5000). AcqKnowledge 4.1 software is used to extract one EEG power every 30 s as absolute power. The 5-minute absolute power at the beginning and end of driving is deleted, SPSS 20.0 software and the method of Pauta criterion are used to remove the abnormal value of EEG power [16], and finally, the analysis of EEG power within 130 minutes is determined.

## 3. Results

### 3.1. Determination of the Fatigue Factor

The absolute power magnitude of the EEG signal varies greatly (as shown in Figure 1). The EEG power of each subject is normalized according to the formula [17], and an average value is taken every five minutes to average the EEG power of 22 drivers. The results are shown in Figure 2. Among them, 30 minutes ago, the change rule was the same, and there were differences among the three wave patterns in 30–130 minutes. The related research shows that the power of *α* and *θ* increases with the increase of fatigue, the increase of *β*-power indicates the increase of alertness, and the larger the ratio of fast wave to slow wave is, the deeper the fatigue is [18, 19]. Therefore, the accumulation rule of fatigue with time shows strong time characteristics. In order to obtain the fatigue factors with obvious time characteristics and strong representativeness, dimension reduction is carried out [20].

SPSS 20.0 and OriginPro 2019 software are used to analyze the five indicators [21]. The results are shown in Figure 3 and Table 3. Autoencoder dimension reduction is shown in Figure 4.

As shown in Figure 3, the coordinate axis and the long and short axis of the confidence ellipse are parallel, indicating that the variable of the long axis describes the main change of the data, and the variable of the short axis describes the secondary change of the data [22]. The characteristic value shows that *F*_1_ represents 3.686 times of the original data, *F*_2_ represents 1.135 times of the original data, and the cumulative percentage of them is 96.42%, which can explain the fatigue rule represented by five indicators [23]. Similar to the principal component analysis (PCA), we also use the autoencoder to provide visual analysis on the two feature dimensions, and the relationship of the power of *α*, *β*, and *θ* is also given accordingly. Expressions (2) and (3) of the main fatigue factor *F*_1_ and the secondary fatigue factor *F*_2_ are derived from the linear relationship between the main components and variables. The change rule of fatigue factors *F*_1_ and *F*_2_ with time is shown in Figure 5 [24].

The larger the fatigue factor is, the deeper the fatigue degree is. The smaller the fatigue factor is, the shallower the fatigue degree is. There is no physiological significance for positive and negative factors [25].

(2) $$\begin{array}{c} F_{1}=0.931\theta +\frac{0.99\theta }{\alpha +\beta }+\frac{0.975\theta }{\alpha }+\frac{0.923\theta }{\beta }-0.189\frac{\alpha }{\beta }, \end{array}$$

(3) $$\begin{array}{c} F_{2}=-0.079\theta +\frac{0.081\theta }{\alpha +\beta }-\frac{0.164\theta }{\alpha }+\frac{0.367\theta }{\beta }+0.98\frac{\alpha }{\beta }. \end{array}$$

### 3.2. Clustering of Fatigue Factors and Determination of High-Fatigue Time

In order to describe the stage characteristics of fatigue, *K*-means test was used to cluster *F*_1_ and *F*_2_. According to the trend analysis of Section 2.1, *F*_1_ and *F*_2_ were clustered into three categories (I and IV, II and V, and III and VI, in which the fatigue degree ranked I < II < III, IV < V < VI, but I, II, III and IV, V, VI had no statistical relationship) [26]. The results are shown in Figure 6.

In order to quantitatively describe the rule of fatigue factor and time, regression analysis is used to fit *F*_1_ with logistic, and the results are shown in Figure 7 and Table 4. According to Figure 5, the fatigue state in 130 min can be divided into two stages: 5–85 min and 90 min–130 min (one EEG average value is taken every 5 min, which represents the EEG power in 5 min. In this paper, the time point at the end of every 5 min represents the EEG power in this period) [27]. In 5–85 min, class I *F*_1_ is dominant, class II *F*_1_ only accounts for 17.65%, and class II and class III *F*_1_ alternate in 90 min–130 min, which account for the same proportion. It can be seen that the driver's fatigue accumulates and fluctuates greatly in 90–130 min. Further sine fitting is carried out for the fatigue factor *F*_1-1_ (100–130 min) in this time, and the results are shown in Tables 3 and 5. Although 90 min and 95 min belong to class II, they are quite different and have no statistical significance, so they are not fitted. *F*_1_ logistic fitting is shown in Figure 7. *F*_1_ sine fitting is shown in Figure 8 [28].

In the same way, Gauss fitting is carried out for *F*_2_, and the results are shown in Figure 9 and Table 5. The overall fatigue state is divided into three stages: 5–65 min, 70–85 min, and 90–130 min [29]. In 5–65 min, *F*_2_ completely belongs to category IV, in 70–85 min, there are two categories V and VI, and the peak value appears in 80 min. In 90–130 min, category IV and category V *F*_2_ alternately appear and share the same proportion. It can be seen that the driver fatigue accumulates and fluctuates greatly in 90–130 min. Furthermore, 70–85 min and 90–130 min were fitted. The results are shown in Figures 10 and 11 and Table 4 [30].

In addition, the time corresponding to the extreme point is the high-fatigue period. According to the application scope of each function, the high-fatigue period of *F*_1_ tends to the end of the driving task; the high-fatigue period of *F*_1-1_ is 106.47 min and 124.47 min; the high-fatigue period of *F*_2-1_ is 79 min; the high-fatigue period of *F*_2-1_ is 80 min; the high-fatigue period of *F*_2-2_ is 104.13 min and 123.17 min. Among them, *F*_1-1_ and *F*_2-2_ were the same for 105 min and 125 min, while *F*_2_ and *F*_2-2_ indicate that the fatigue factor fluctuates greatly in 70–85 min and peaks at 80 min. At this time, the *F*_1_ fitting curve in Figure 7 shows a significant inflection point and the trend of sudden increase. It can be seen that 70–85 min is the transition stage from the driver to the fatigue state [31]. Therefore, fatigue can be divided into three stages: 5–65 min no fatigue stage, 70–85 min fatigue transition stage, and 90–130 min fatigue stage. *F*_2-1_ Gauss fitting is shown in Figure 10.

### 3.3. Fatigue Variation with Time

Based on the above analysis, the driver fatigue shows significant time characteristics. There is no obvious fatigue accumulation within 5–65 minutes, and the fatigue factor fluctuates in a small range. Each increase and decrease is controlled within 10 minutes. The driver's fatigue regulation mechanism can completely prevent the accumulation of fatigue on the time axis. The specific rule is *F*_1_ and *F*_2_ decrease within 5–10 min, the driving task is just started, the driver needs to adapt to the driving task, fbe concentrated with full of freshness to the environment, and should not show a negative mental state of fatigue. Within 15–65 minutes, the driver's mental state is stable, even though *F*_1_ fluctuates slightly, but fatigue does not accumulate with time. *F*_2-2_ sine fitting is shown in Figure 11.

In 70–85 min, *F*_2_ showed a significant Gauss wave pattern. The significant peak appeared at 80 min, and the recovery period from the peak appeared to 15 min.

In 90–130 minutes, *F*_1_ and *F*_2_ showed a significant sine wave pattern. *F*_1-1_ fluctuates periodically in 9 min and *F*_2_ in 9.52 min. At the same time, the peak value of the two increases. It can be seen that although the driver's fatigue regulation ability can play a role, fatigue still increases with time. From the analysis of Section 2.2, it is known that the fit of *F*_1_ and *F*_2_ for the high-fatigue period is only 2.34 min, within 5 min, and the gap tends to decrease, so it is more reasonable to use the secondary fatigue factor *F*_2_ to describe the rule of the fatigue transition stage and fatigue stage. The fatigue model of the grassland road driver is summarized as the following formula:

(4) $$\begin{array}{c} F=\left\{\begin{array}{c} 1.22+1.62e^{-1.06{\left(t-80\right)}^{2}},70\leq x\leq 85,\\ 0.3+\sin\left[\left(\frac{t-1.37}{9.5}\right)\pi \right],90\leq x\leq 130. \end{array}\right. \end{array}$$

### 3.4. The Classification Accuracy in Driving Fatigue Detection

Table 4 summarizes the classification accuracy in driving fatigue detection as achieved by the six classification models for each subject. The results show that our model classifier achieves the highest accuracy for all the subjects in classifying the fatigue vs. alert states. Our model achieves higher accuracy and yields lower variance than the RBF-ROLS + D-opt network. This shows that among these two RBF-based classifiers, the EEG driving fatigue detection proposed in this paper is a more accurate and robust classifier.

Compared to the other models, our model exhibits the best performance regardless of the specificity, sensitivity, and accuracy. In addition, the RBF-TLLH model significantly outperforms the RBF-ROLS + D-opt model in sensitivity, demonstrating the superiority of the proposed approach to detect driving fatigue. Compared to RBF-ROLS + D-opt, the proposed RBF-TLLH model achieves a slightly lower specificity, but a much higher accuracy and sensitivity.

## 4. Discussion

1. The conclusion shows that the driver enters the fatigue stage obviously after 90 minutes. Although the fatigue factor increases and fluctuates greatly, the peak increase of the sine wave is small. Up to now, there is no clear division of light, medium, and heavy fatigue in the world. Because the driving task in this paper is only 130 minutes, there is no comparison between other types of fatigue, and it can only be defined as fatigue. As for the fatigue level, it is true that it is necessary to arrange long-term driving tasks for comparative study.
2. 70–85 min is the transition period from the driver to fatigue. According to *F*_2_ interpretation, the rule changes with the sine function after 80 min peak, and each cycle of fatigue and recovery is 9.52 min; according to *F*_1_ interpretation, 70–85 min does not show fatigue, and it suddenly increases within 85–100 min, from which fatigue begins to accumulate. The derivative of *F*_1_ in 85–110 min is analyzed, as shown in Figure 11; the derivative is 37 times of the derivative of 85 min, which is similar to the mutation rule characterized by *F*_2_ in 70–85 min. The mutation period is 15 min at the same time, and *F*_2_ is mutated before *F*_1_. It is confirmed that the transition from the fatigue-free stage to fatigue stage needs to be completed by mutation and recovery of the fatigue factor, but it is impossible to determine that *F*_1_ mutation lags behind *F*_2_. The analysis of the change rule of the fatigue transition period is of guiding significance for the measures to prevent the formation of fatigue. Therefore, a large number of experimental samples are needed to study the change rule of the fatigue transition period.
3. For the fatigue prediction after 100 min, the sine wave function of *F*_1_ and *F*_2_ has a high fitting degree, with a period difference of 0.52 min (see Figure 11). At first, the peak value corresponds to a time difference of 1/4 sine cycles, *F*_2_ is earlier than *F*_1_, but because of the long period of *F*_2_, *F*_1_ will reach the peak value at *t* = 142.47 min and *F*_2_ will reach the peak value at *t* = 142.21 min with the increase of time; at this time, *F*_1_ and *F*_2_ change rule coincide. Later, if *F*_1_ and *F*2 still meet the current sine function law, they will fluctuate according to the superposition sine wave law. The peak value of *F*_1_ is 0.76 min earlier than that of *F*_2_. According to the superposition principle of wave, at this time, fatigue will accumulate to a higher peak value in the time-axis direction, indicating the deepening of fatigue. Due to the limited time of driving tasks in this paper, the driving fatigue after 100 minutes cannot be determined, only the effect can be predicted, and large samples and simulation experiments are needed to arrange long-term driving tasks for further explanation.

## 5. Conclusions

In this paper, we propose an ant colony optimization algorithm based on mobile sink data collection in industrial wireless sensor networks. The fatigue factors are determined as *F*_1_=0.931*θ*+(0.99*θ*/*α*+*β*)+(0.975*θ*/*α*)+(0.923*θ*/*β*) − (0.189*α*/*β*) and *F*_2_=−0.079*θ*+(0.081*θ*/*α*+*β*) − (0.164*θ*/*α*)+(0.367*θ*/*β*)+(0.98*α*/*β*).

*F*_1_ and *F*_2_ contain 96.42% EEG power information of fatigue changing with time during 130 min driving. Through regression analysis, *F*_1_ and *F*_2_ together show that the high incidence time of driving fatigue is 105 min and 125 min. The change of driving fatigue with time can be divided into three stages: 5–65 min is the nonfatigue stage, 70–85 min is the fatigue transition stage, and 90–130 min is the fatigue stage. The variation of fatigue with time obeys function expression (4).

## Figures and Tables

**Figure 1:** Absolute power (*α*, *β*, and *θ*) of 6 drivers.

**Figure 2:** Changes in the EEG relative power of 22 drivers over time.

**Figure 3:** Principal component analysis confidence ellipses for 5 indicators.

**Figure 4:** Autoencoder dimension reduction.

**Figure 5:** Driver fatigue factor changes with time.

**Figure 6:** Cluster analysis results.

**Figure 7:** *F*_1_ logistic fitting.

**Figure 8:** *F*_1-1_ sine fitting.

**Figure 9:** *F*_2_ Gauss fitting.

**Figure 10:** *F*_2-1_ Gauss fitting.

**Figure 11:** *F*_2-2_ sine fitting.

**Table 1:** Subject information.

Gender	Number	Age	Driving age	BIM
Female	6	32.51 ± 5.23	3.12 ± 1.33	19.53 ± 5.42
Male	24	35.46 ± 7.47	3.97 ± 2.29	21.59 ± 2.77

**Table 2:** Statistics of relevant parameters for the S101 section line.

Speed limit	Line type						Landscape		
80 km/h	Route length (km)	The longest straight line (m)	Linear density (km/km)	Maximum curve radius (m)	Curve radius distribution (m) and proportion (%)	Maximum longitudinal grade (%)	Desertification is serious (%)	Medium vegetation coverage (%)	High vegetation coverage (%)
	150	8741	0.849	40,000	1000–2000/61	−4.92	13	67	20

**Table 3:** Principal component analysis results.

	The total variance of the principal components		Component matrix				
	Characteristic value	Cumulative percentage (%)	*θ*	*θ*/(*α*+*β*)	*θ*/*α*	*θ*/*β*	*α*/*β*
*F*_1_	3.686	73.728	0.931	0.990	0.975	0.923	−0.189
*F*_2_	1.135	96.419	−0.079	0.081	−0.164	0.367	0.980

**Table 4:** The accuracy of classification results.

Classification matrix	Model					
	ANN-BP (%)	ANN-PSO (%)	RBF-ROLS + D-opt (%)	[32] (%)	[33] (%)	Our model (%)
Sensitivity/TPR	76.67	71.81	80.00	92.36	82.36	93.26
Specificity/TNR	76.94	62.78	95.56	93.06	83.09	92.78
Accuracy (%)	76.81	67.29	87.78	86.98	85.72	90.07

**Table 5:** Fitting formula and fitting degree.

Fitting formula	Adj. *R*^2^	*t*	*dF*/*dt*=0
*F*_1_=1.21 − (1.77/1+(0.01*t*)^40.94^)	0.61>0.4	5–130	*t*⟶+*∞*
*F*_1−1_=1.2+sin[(*t*+6.03/9)*π*]	0.48>0.4	100–130	*t* = −1.53±9*k*, *k* = 0, 1, 2, 3⋯
*F*_2_=−0.29+2.83*e*^−0.02(*t* − 79)^2^^	0.45>0.4	5–130	79
*F*_2−1_=1.22+1.62*e*^−1.06(*t* − 80)^2^^	1.00 > 0.4	70–85	80
*F*_2−2_=0.3+sin[(*t* − 1.37/9.5)*π*]	0.80>0.4	90–130	*t* = 18.45±9.52*k*, *k* = 0, 1, 2, 3⋯

## Data Availability

All the data used to support the findings of this study are available from the corresponding author upon request.

## References

[1] Thiffault P., Bergeron J. (2003). Fatigue and individual differences in monotonous simulated driving. *Personality and Individual Differences*.

[2] Thiffault P., Bergeron J. (2003). Monotony of road environment and driver fatigue: a simulator study. *Accident Analysis & Prevention*.

[3] Oron-Gilad T., Ronen A., Shinar D. (2008). Alertness maintaining tasks (AMTs) while driving. *Accident Analysis & Prevention*.

[4] Lal S. K. L., Craig A. (2001). A critical review of psychophysiological of driver fatigue. *Biological Psychology*.

[5] Larue G. S., Rakotonirainy A., Pettitt A. N. (2011). Driving performance impairments due to hypovigilance on monotonous roads. *Accident Analysis & Prevention*.

[6] Fell D. L., Black B. (1997). Driver fatigue in the city. *Accident Analysis & Prevention*.

[7] Pollock V. E., Schneider L. S., Lyness S. A. (1991). Reliability of topographic quantitative EEG amplitude in healthy late-middle-aged and elderly subjects. *Electroencephalography and Clinical Neurophysiology*.

[8] Fletcher L., Petersson L., Zelinsky A. Road scene monotony detection in a fatigue management driver assistance system.

[9] Larue G. S., Rakotonirainy A., Pettitt A. N. (2011). Driving performance impairments due to hypovigilance on monotonous roads. *Accident Analysis & Prevention*.

[10] Li W., He Q. C., Fan X. M., Fe Z. M. (2011). Study on driving fatigue of grassland highway based on EEG signal. *Neuroscience Letters*.

[11] Abojaradeh M., Jrew B., Ababsah H. (2014). Study on driver’s driving characteristics and road traffic safety countermeasures. *Transportation and Engineering*.

[12] Phillip P., Taillard J., Klein E. (2003). Experimental Study on fatigue accumulation of long-distance bus drivers. *Journal of Psychosomatic Research*.

[13] Huang H., Zhang F., Yu L. Overview of non-contact pantograph-catenary arc detection based on image processing.

[14] Gillberg M., Kecklund G., Åkerstedt T. (1996). Sleepiness and performance of professional drivers in a truck simulator - comparisons between day and night driving. *Journal of Sleep Research*.

[15] Wascher E., Arnau S., Gutberlet I., Karthaus M., Getzmann S. (2018). Evaluating Pro- and Re-active driving behavior by means of the EEG. *Frontiers in Human Neuroscience*.

[16] Zhao X., Wei Z., Li Z., Zhang Y., Feng X. (2015). Threshold research on highway length under typical landscape patterns based on drivers’ physiological performance. *Discrete Dynamics in Nature and Society*.

[17] Ahn S., Nguyen T., Jang H., Kim J. G., Jun S. C. (2016). Exploring neuro-physiological correlates of drivers’ mental fatigue caused by sleep deprivation using simultaneous EEG, ECG, and fNIRS data. *Frontiers in Human Neuroscience*.

[18] Bastien C. H., Ladouceur C., Campbell K. B. (2000). EEG characteristics prior to and following the evoked K-Complex. *Canadian Journal of Experimental Psychology*.

[19] Lal S. K. L., Craig A., Boord P., Kirkup L., Nguyen H. (2003). Development of an algorithm for an EEG-based driver fatigue countermeasure. *Journal of Safety Research*.

[20] Zhao T., Qi C., Zhu S. (2016). Study on multi index division of short-term driving fatigue of grassland highway. *Chinese Journal of safety Sciences*.

[21] Chen C. H., Song F., Hwang F. J, Wu L. (2020). “A probability density function generator based on neural networks. *Physica A: Statistical Mechanics and its Applications*.

[22] Farias G. D. J., Savian J. V. (2020). Integrated crop-livestock system with system fertilization approach improves food production and resource-use efficiency in agricultural lands. *Agronomy for Sustainable Development*.

[23] Kumar A., Bawa S. (2020). DAIS: dynamic access and integration services framework for cloud-oriented storage systems. *Cluster Computing*.

[24] Nandi M. L., Nandi S., Moya H., Kaynak H. (2020). Blockchain technology-enabled supply chain systems and supply chain performance: a resource-based view. *Supply Chain Management: International Journal*.

[25] Sahoo S. S., Nguyen T., Veeravalli B. (2019). Multi-objective design space exploration for system partitioning of FPGA-based Dynamic Partially Reconfigurable Systems. *Integration*.

[26] Sharma T., Balachandra P. (2019). Model based approach for planning dynamic integration of renewable energy in a transitioning electricity system. *International Journal of Electrical Power & Energy Systems*.

[27] Roekel H., Steen M. (2019). Integration as unrealised ideal of ERP systems: an exploration of complexity resulting from multiple variations of integration. *Qualitative Research in Accounting and Management*.

[28] Zhang L., Pu J. An improved back propagation neural network in objects recognition.

[29] Li C., Liu X. An improved PSO-BP neural network and its application to earthquake prediction.

[30] Chen S., Hong X., Harris C. (2003). Sparse kernel regression modeling using combined locally regularized orthogonal least squares and D-optimality experimental design. *IEEE Transactions on Automatic Control*.

[31] Ren Z., Li R., Chen B. (2021). EEG-based driving fatigue detection using a two-level learning hierarchy radial basis function. *Frontiers in Neurorobotics*.

[32] Wang F., Wu S., Ping J., Xu Z., Chu H. (2021). EEG driving fatigue detection with PDC-based brain functional network. *IEEE Sensors Journal*.

[33] Karakose E., Gencoglu M. T., Karakose M., Yaman O. (2018). A new arc detection method based on fuzzy logic using S-transform for pantograph‐catenary systems. *Journal of Intelligent Manufacturing*.

